# Nursing Effect and Prognosis Analysis of Self-Management Education Model Based on Protective Motivation Theory on Patients with Hematological Tumor after PICC Catheterization

This article has been retracted.

**DOI:** 10.1155/2022/4180113

**Published:** 2022-05-13

**Authors:** Lili Jiang, Xiuying Yang, Lu Xi, Chaolang Zhang

**Affiliations:** Department of Hematology-Oncology, The Children's Hospital, Zhejiang University School of Medicine, Pediatric Leukemia Diagnostic and Therapeutic Technology Research Center of Zhejiang Province, National Clinical Research Center for Child Health, Hangzhou 310000, China

## Abstract

**Objective:**

To analyze the nursing effect and prognostic value of self-management education model based on protective motivation theory on patients with hematological malignancies (HM) after peripheral venous catheterization (PICC).

**Methods:**

A total of 90 patients with HMs treated with PICC catheterization in our hospital from October 2019 to October 2021 were included in the study. The patients were randomly assigned into experimental group (*n* = 45) and control group (*n* = 45). On the basis of the control group, the experimental group implemented the self-management education model based on the theory of protective motivation, and the control group implemented routine nursing health education measures. The self-nursing ability scale (ESCA), Hamilton anxiety scale (HAMA), the average cost of PICC catheter maintenance, the incidence of PICC-related complications, and the score of Newcastle nursing satisfaction scale (NSNS) were observed 1 month before and after nursing.

**Results:**

After one month of nursing, there was no significant difference in ESCA self-concept (*p* > 0.05). After one month of nursing, the scores of self-care responsibility, self-nursing skills, and health knowledge in the experimental group were significantly higher compared to those before nursing (*p* < 0.05) and higher compared to those in the control group (*p* < 0.05). After one month of nursing, the score of HAMA scale was significantly lower compared to that before nursing (*p* < 0.05), and the score of HAMA scale in the experimental group was lower compared to the control group (*p* < 0.05). After one month of nursing, the average cost of PICC pipeline maintenance in the test group was lower than that in the control group (*p* < 0.05). One month after nursing, the incidence of PICC-related complications in the experimental group was lower than that in the control group (*p* < 0.05). One month after nursing, the score of NSNS scale was significantly higher than that before nursing (*p* < 0.05). After one month of nursing, the score of NSNS scale in the experimental group was higher than that in the control group.

**Conclusion:**

The self-management education model based on protective motivation theory is effective in nursing patients with peripheral venous catheterization and PICC catheterization of HMs. It is more beneficial to promote patients' self-nursing management ability, reduce anxiety, reduce the average cost of PICC pipeline maintenance, reduce the incidence of PICC-related complications, and enhance nursing satisfaction.

## 1. Introduction

Hematological malignancies (HM), defined as a hematological malignant tumor, refers to a malignant clonal disease originating from the hematopoietic system, which occupies the sixth place in the incidence of all tumors [1]. The incidence rate in China is 2.76/100000 [2]. As we all know, intravenous chemotherapy is an indispensable part of comprehensive treatment of HMs. However, it is common for chemotherapeutic drugs to damage blood vessels because of their chemical properties, acidity, alkalinity, and high concentration. Peripherally inserted central venous catheter (PICC) refers to the technique of deep venous catheterization from the peripheral vein and the end of the catheter to the central vein [3]. In terms of the traditional drug administration, such as subclavian vein administration and jugular vein administration, it has the advantages of convenient operation, high safety, long-term use, and reduction the vascular damage caused by repeated venipuncture and chemotherapeutic drugs or hypertonic fluid [4]. Although PICC can greatly solve the problem of vascular injury and repeated puncture pain in tumor patients during chemotherapy, the coagulation function of HM patients is poor, and they are more likely to have complications such as puncture point bleeding, mechanical phlebitis, venous thrombosis, puncture point infection, low immunity, and bone marrow suppression after chemotherapy. Studies have shown that the incidence of PICC complications can be as high as 30.9%, and catheter-related complications may occur at any time in the process of PICC catheterization [5]. Regarding other stages, PICC catheter-related complications are more likely to occur within one month after catheterization. The length of catheterization time is related to nurses, patients, and their families' knowledge of daily maintenance of PICC and the ability of self-management of PICC catheterization, especially the understanding of PICC complications and related to correct management [6].

American nursing expert Orem put forward the concept of self-care in 1971 [7]. In 1990, Gantz further proposed that self-nursing can be assigned into two parts: self-nursing maintenance and self-nursing management [8]. Self-care maintenance refers to following correct health behaviors, such as proper diet, proper exercise, and taking medicine as directed by a doctor; self-care management includes a series of comprehensive and complex processes such as identifying subtle changes in one's health, assessing the importance of symptoms and signs, correctly dealing with symptoms and signs, and monitoring the effectiveness of treatment [9]. The related studies have indicated that the self-management behavior of tumor patients plays a key role in the prevention and control of PICC complications, so the self-management of PICC catheter has become the key of the management of patients with PICC catheterization [10]. The theory of protective motivation was put forward by Rogers and other scholars [11]. The theory explains the process of behavior change through threat assessment and coping assessment in the process of cognitive regulation and discusses the formation of healthy behavior from motivational factors [12]. With the further development of protective motivation theory, this theory has been widely used in patients with duodenal ulcer, percutaneous coronary intervention, and the improvement of self-management ability of postoperative rehabilitation patients with thoracolumbar burst fracture [13]. Therefore, a total of 90 patients with HM treated with PICC catheterization in our hospital from October 2019 to October 2021 were included in this experiment to analyze the nursing effect and prognostic value of self-management education model based on protective motivation theory on HM patients with PICC catheterization, in order to better meet the needs of patients and provide new ideas for clinical nursing research of HM patients with PICC catheterization [14].

## 2. Patients and Methods

### 2.1. General Information

A total of 90 patients with HMs treated with PICC catheterization in our hospital from October 2019 to October 2021 were included in the study. The patients were randomly assigned into experimental group (*n* = 45) and control group (*n* = 45). The inclusion criteria were as follows: (1) patients diagnosed as HMs by clinical examination; (2) first chemotherapy and placement of PICC catheter; (3) patients aged more than 18 years old, primary school education and above, with certain reading comprehension ability; and (4) conscious, informed consent, and voluntary participation in this study. Exclusion criteria were as follows: (1) patients who did not support or cooperate with tumor chemotherapy in this study, (2) patients with superior vena cava syndrome and severe hemorrhagic diseases that were not suitable for catheterization, and (3) severe hearing and visual impairment.

### 2.2. Treatment Scheme

Patients were treated with Bard's three-way valvular PICC catheter (see Figures 1(a) and 1(b)), model 4Fr, ultrasound-guided Sedinger technique, and needle-free infusion connector (BD separator) made by BD Company. The catheter is maintained using a disposable central venous catheterization maintenance kit from Asia and Australia and a 10 ml prefilled syringe from BD.

For the scheme of the reference group, routine nursing health education measures were implemented. The main results were as follows: (1) before catheterization, the PICC specialist nurse explained to the patients the matters needing attention during catheterization, the complications related to PICC, and the possible adverse events during catheterization, and the PICC assistant explained the relevant precautions and cooperative actions to the patients in the process of catheterization; (2) after catheterization, PICC specialist nurses could improve the catheter awareness of patients with catheters by recommending health education videos related to PICC or issuing health manuals. Responsible nurses need to communicate with patients one-to-one every day, publicize, evaluate the local situation of patients with catheterization, timely feedback, and write records; (3) after discharge, the patients with tube were followed up by telephone according to the routine. The frequency was 1 to 2 times per month, keeping 10 min/time, in order to understand the current situation of PICC management of patients with tube.

For the scheme of the experimental group, on the basis of the reference group, the self-management education model based on the theory of protective motivation was implemented. The details are shown in Table 1.

### 2.3. Observation Index

1. To observe the score of ESCA before nursing and 1 month after nursing, the ESCA scale included 4 items and 43 items, including self-concept (8 items), sense of self-care responsibility (6 items), self-care skills (12 items), and health knowledge level (17 items). The scale was scored with a scale of 0-4 points and 5 levels, including 4 points: very much like me; 3 points: a little like me; 2 points: uncertain; 1 point: some are not like me; 0 points: very unlike me. The total score was 172. The higher the score, the stronger the self-care ability
2. The scores of HAMA were observed before nursing and 1 month after nursing. The score of HAMA < 7 means that the patient has no anxiety; the score is from 7 to 13 representing the possibility of anxiety; the score is from 14 to 20 indicating that the patient must have anxiety; the score ranges from 21 to 28 indicating that the patient has obvious anxiety; the score ≥ 29 indicates that the patient's anxiety is serious
3. The average cost of PICC pipeline maintenance was observed after 1 month of nursing
4. The incidence of PICC-related complications was observed after one month of nursing. Possible PICC-related complications include phlebitis, percolation at the puncture point, catheter blockage, skin allergy, venous thrombosis, and catheter prolapse
5. The scores of Newcastle NSNS were observed before nursing and 1 month after nursing. A total of 19 test projects ((1) the time how long the nurse spent on you; (2) the working ability of nurses; (3) when you need it, there will always be a nurse by your side. The nurse's understanding of your situation; (5) the speed at which they come when you call the nurse; (6) the way the nurses treat you makes you feel at home; (7) the amount of information that nurses provide you with diseases and treatments; (8) the number of times nurses checked the ward; (9) the help provided by the nurse; (10) the way the nurse explains the problem for you; (11) the extent to which the nurse reassured your relatives or friends; (12) nurses' attitude towards their own work; (13) the type of confidence that nurses provide you with diseases and treatment; (14) the nurse's respect for you in the course of nursing; (15) the way nurses listen to your troubles and concerns; (16) under the premise of abiding by the rules and regulations, the degree of freedom given to you by the nurse during hospitalization; (17) the nurse's willingness to respond to your request; (18) the degree of protection of your privacy by nurses; (19) nurses can understand your needs), the total score ranges from 0 to 95. Each item was evaluated with a score of 1 to 5, of which 1 is very dissatisfied, 2 is dissatisfied, 3 is general satisfaction, 4 is satisfied, and 5 is very satisfied. The higher the score, the higher the satisfaction

### 2.4. Statistical Analysis

The statistical analysis of the data in this study uses the SPSS 24.0 software, and the statistical graphics are drawn by GraphPad Prism 8.0. The measurement data in accordance with normal distribution were presented by mean ± standard deviation ($\overset{-}{x}\pm S$), paired sample *t*-test was employed for intragroup comparison, and independent sample *t*-test was employed for intergroup comparison (*p* < 0.05). If not, it was presented by median (lower quartile to upper quartile), paired sample nonparametric test was employed for intragroup comparison, and independent sample nonparametric test was employed for intergroup comparison. The grade data were tested by FISHER accurate method. *p* < 0.05 was exhibited statistical significance.

## 3. Results

### 3.1. The Score of ESCA Scale before Nursing and 1 Month after Nursing

There was no significant difference in ESCA self-concept after one month of nursing. One month after nursing, the scores of self-care responsibility, self-care skills, and health knowledge in the experimental group were significantly higher than those before nursing (*p* < 0.05) and higher compared to the control group (*p* < 0.05), as indicated in Tables 2–5.

### 3.2. The Score of HAMA Scale before Nursing and 1 Month after Nursing

One month after nursing, the HAMA score was significantly lower than that before nursing (*p* < 0.05). After one month of nursing, the score of HAMA scale in the experimental group was lower than that in the control group, as indicated in Table 6.

### 3.3. The Average Cost of PICC Pipeline Maintenance before and 1 Month after Nursing

After one month of nursing, the average cost of PICC pipeline maintenance in the experimental group was lower compared to the control group (*p* < 0.05), as indicated in Table 7.

### 3.4. The Incidence of PICC-Related Complications after One Month of Nursing

After one month of nursing, the incidence of PICC-related complications in the experimental group was lower compared to the control group (*p* < 0.05), as indicated in Table 8.

### 3.5. The Score of NSNS Scale before Nursing and 1 Month after Nursing

After one month of nursing, the scores of NSNS scale were significantly higher compared to those before nursing (*p* < 0.05). After one month of nursing, the score of NSNS scale in the experimental group was higher compared to the control group (*p* < 0.05), as indicated in Table 9.

## 4. Discussion

PICC was introduced into clinic as a way of parenteral nutrition support. In 1990s, this technology was introduced into China [15–19]. Because the head of the PICC catheter is located in the central vein and has a large blood flow, it can quickly reduce the liquid osmotic pressure and drug concentration and reduce the risk of recurrent puncture pain, phlebitis, and peripheral vascular necrosis caused by exudation of chemotherapeutic drugs [20, 21]. Although PICC can greatly solve the problem of vascular injury and repeated puncture in tumor patients undergoing chemotherapy, it is easy to affect the compliance of daily catheter maintenance, resulting in an increase in the incidence of PICC complications, not only inconvenience to patients but also increased out-of-hospital maintenance costs [22–24]. Health education is an effective way to strengthen self-care. The theory of protective motivation is an important theory to track and explore the formation principle behind behavior. The mechanism is that the subject evaluates himself in order to take positive actions to deal with threats, reduce the risk of unhealthy behaviors, and promote the establishment of healthy behaviors [25]. Therefore, the purpose of this study is to analyze the nursing effect and prognostic value of self-management education model based on protective motivation theory on hypertensive patients with PICC catheterization, in order to find a more effective health education and nursing program.

The results of our study indicated that one month after receiving the self-management education model based on protective motivation theory, the scores of ESCA self-care responsibility, self-nursing skills, and health knowledge were significantly higher than those before nursing (*p* < 0.05) and higher than those of routine health education (*p* < 0.05). It is proved that the self-management education model based on protective motivation theory is more helpful to improve the self-nursing ability of HM patients with PICC catheterization. This is mainly because, according to the theory of protective motivation, a number of intervention measures such as health education, face-to-face interviews, scenario simulation, and deliberate practice are comprehensively used to strengthen patients' understanding of the seriousness and possibility of improper management of PICC, weaken the internal and external rewards for patients to form bad health behaviors, reduce patients' reaction costs, and stimulate patients' behavior motivation [26]. On the other hand, in the process of health intervention, we should not only pay attention to the strengthening of patients' knowledge related to PICC catheter, make them effectively master the necessary knowledge and skills of PICC catheter self-management, and increase patients' catheter cognitive level, catheter management ability, and confidence but also make patients actively aware of their own problems and overcome the oneness of nurses as the main body of the traditional health education model [26, 27].

One month after receiving the self-management education model based on protective motivation theory, the HAMA score of patients was lower compared to routine health education (*p* < 0.05). It is proved that the self-management education model based on protective motivation theory is more helpful to alleviate the anxiety of patients with HM after PICC catheterization. This is mainly because patients with malignant HMs have a long course of disease, and in the process of PICC catheterization chemotherapy [23], they will worry about the side effects of chemotherapy and the prognosis of the disease and often have anxiety and fear [24]. Lack of catheter-related knowledge, worry about catheter maintenance after discharge, and possible complications are important causes of bad mood [25]. The self-management education model based on protective motivation theory not only carries out health education to patients but also teaches the knowledge and skills of self-nursing, which not only enhances the ability of self-management but also increases the degree of attention to patients' treatment, increases patients' confidence in PICC catheterization maintenance, eliminates the worries of inadequate maintenance of PICC catheterization, and alleviates anxiety symptoms.

One month after receiving self-management education model based on protective motivation theory, the average cost of PICC pipeline maintenance was lower compared to routine health education. The score of NSNS scale was higher than that of routine health education. It is proved that the self-management education model based on protection motivation theory is more helpful to reduce the maintenance cost of PICC pipeline and promote patient satisfaction. This is mainly because PICC can avoid the pain of repeated puncture and the harm caused by chemotherapeutic drugs to venous stimulation, but the cost of catheter maintenance in hospital cannot be ignored [26]. Some studies have indicated that medical expenses and round-trip transportation time are the main factors affecting satisfaction [27]. With the extension of travel time, the travel fare increases, and satisfaction decreases significantly. Through self-management education based on protective motivation theory, patients and their families master the methods of keeping PICC effective and unobstructed, learn to take self-care of catheters, establish a regular lifestyle, avoid the trouble when coming to the hospital every week for maintenance, facilitate patients, reduce their financial burden, prolong the indwelling time of catheters, ensure continuous treatment of chemotherapy, and bring practical benefits and convenience to patients.

One month after receiving the self-management education model based on protective motivation theory, the incidence of PICC-related complications was lower than that of routine health education (*p* < 0.05). It is proved that the self-management education model based on protective motivation theory is more helpful to reduce the incidence of PICC-related complications. This is mainly because, through the self-management education of protective motivation theory, patients have mastered certain PICC-related knowledge and management skills [26]. They are aware of their dominant position in the process of PICC management and the late clinical nursing difficulties and economic losses caused by catheter prolapse, form relatively healthy behavior habits, and always keep relevant precautions and operating skills in mind in daily life and activity exercise. In addition, in the process of intervention, this study focuses on weakening the internal and external rewards that lead to patients' bad habits, while emphasizing the important attributes of family members in the process of PICC management, encouraging patients' family members to participate in the process, and by empowering patients' family members to change the form of passive acceptance and simple repetition, so as to stimulate the initiative of patients' family members to learn to take care of them and enhance the self-efficacy [27].

In summary, the self-management education model based on protective motivation theory is effective in nursing patients with peripheral venous catheterization and PICC catheterization of HM. It is more helpful to promote patients' self-nursing management ability, reduce anxiety, reduce the average cost of PICC pipeline maintenance, reduce the incidence of PICC-related complications, and enhance nursing satisfaction. There are some limitations in this study. First of all, the sample size of this study is small, and it is a single-center study, so the results of the study are inevitably biased. In future research, we will expand the sample size and carry out multicenter prospective studies, which may lead to more valuable conclusions.

## Figures and Tables

**Figure 1:** (a) Screenshot of PICC tube placement DVD (courtesy of Bard). (b) Screenshot of PICC tube placement DVD (courtesy of Bard).

**Table 1:** The specific content of self-management education based on the theory of protective motivation.

Time	Specific content
The day before or after the placement of the tube	(1) Ask the patient to agree on the learning time—before or after catheterization (2) Collect as many multimedia materials, pamphlets, or books related to PICC health education as possible before intervention (3) Choose a relatively quiet and tidy room, the nurse gives a brief self-introduction to the patient to gain the trust of the patient; the patient can invite his family or friends to participate in order to create a relaxed and comfortable communication environment (4) To understand the current situation of patients' knowledge related to PICC self-management in the question-and-answer form (5) Patients are encouraged to choose their favorite way of learning, according to their different perceptual preferences, adopt different forms of education, if for visual learners, choose to use video, pictures, etc., to stimulate them to receive information; if they are auditory learners, then choose audio and other forms for health education. For kinesthetic learners, they are encouraged to understand information by taking notes, drawing charts, or doodling, etc., and carry out open learning based on the theme of improving patients' understanding of the seriousness and susceptibility of improper management of PICC. The intervention time was 20~30 mins

4 days after catheterization	(1) In the form of face-to-face interviews, patients and their families are asked to recall the practice of PICC self-management process during this period, and patients are encouraged to talk about the problems or worries that may exist in the current PICC self-management behavior (such as being afraid to move or excessive activity). Analyze the internal and external causes of this unhealthy behavior, such as asking the patient “what benefits do you think this will bring to you?,” help patients find alternative solutions, and correct the subjective benefit of patients' bad behavior (2) In the process of intervention, we should pay attention to the important value of family members in the self-management of patients' PICC, strengthen the health education to patients' families, and weaken the formation of patients' bad health behavior caused by external factors. The intervention time was 10~15 mins

The seventh day after catheterization	(1) Communicate deeply with the patients and their families, so as to judge the patients' mastery of health information and establish personal files (2) According to the weaknesses of the patients' self-management, the self-management education group plays the corresponding situational simulation video of PICC self-management to explain to the patients the management skills and thinking paths used in the case videos (3) The self-management education team writes a similar script according to the scene presented in the video and asks the patients to conduct situational exercises with each other after writing. After exercise, the patients reflect on themselves, and the members of the group give timely feedback to point out the existing problems and areas for further improvement in the simulation process. The patients conduct situational exercises again; that is, after each round of drills, they conduct drills according to the existing problems and countermeasures of the previous round to consolidate the operation skills. The intervention time was 20~30 mins

From discharge to the fourth week after catheterization	(1) On the day of discharge, set up a WeChat group and pull the patients and their families into the WeChat group. When setting up into the group, you need to go through the verification of the group owner, answer the questions raised by the patients, answer them in time, and reduce the obstacles in the process of PICC self-management during the patient's stay at home (2) With the consent of the patients, the patients are actively followed up twice in the form of remote video during the first intermission of chemotherapy. The contents of the follow-up include the education of PICC self-management knowledge at home, the observation of local skin at the PICC puncture site, and so on. For each 5 ~ 10 mins, the specific time point will be decided after consultation with the patient (if the patient is unable to carry out remote video follow-up, it will be in the form of telephone follow-up) (3) Pay attention to the differences of individual cognitive level caused by various factors among patients, and for patients with low cognitive level, we can deepen their cognition by means of pictures or videos and so on (4) When carrying on the health education to the family members, point out to them the important role they play in the psychology and emotion of the patients, and improve the role sense of the patients' families and the social support to the patients

**Table 2:** ESCA scale-self-concept score was observed before nursing and 1 month after nursing.

ESCA scale-self-concept (score)	Before nursing	After one month of nursing	*t*	*p*
Reference group (*n* = 45)	15.12 ± 1.39	15.19 ± 1.25	0.151	0.802
Test group (*n* = 45)	15.14 ± 1.44	15.23 ± 1.35	0.305	0.760
*t*	0.067	0.145		
*p*	0.946	0.884		

**Table 3:** ESCA scale-self-care responsibility score was observed before nursing and 1 month after nursing.

ESCA scale-sense of self-care responsibility (score)	Before nursing	After one month of nursing	*t*	*p*
Reference group (*n* = 45)	12.45 ± 1.27	16.99 ± 2.07	12.540	<0.001
Test group (*n* = 45)	12.48 ± 1.15	19.32 ± 3.25	13.309	<0.001
*t*	0.117	4.056		
*p*	0.906	<0.01		

**Table 4:** ESCA scale-self-nursing skill score was observed before nursing and 1 month after nursing.

ESCA scale-self-care skills (points)	Before nursing	After one month of nursing	*t*	*p*
Reference group (*n* = 45)	21.78 ± 1.49	30.11 ± 3.18	15.902	<0.001
Test group (*n* = 45)	21.88 ± 1.15	40.05 ± 4.24	27.744	<0.001
*t*	0.356	12.581		
*p*	0.722	<0.01		

**Table 5:** To observe the score of ESCA scale-health knowledge level before and 1 month after nursing.

ESCA scale-level of health knowledge (points)	Before nursing	After one month of nursing	*t* value	*p* value
Reference group (*n* = 45)	32.11 ± 1.25	50.02 ± 2.17	49.684	<0.001
Test group (*n* = 45)	32.17 ± 1.39	61.58 ± 5.11	35.783	<0.001
*t*	0.215	14.065		
*p*	0.830	<0.01		

**Table 6:** To observe the score of HAMA scale before nursing and 1 month after nursing.

HAMA scale score (points)	Before nursing	After one month of nursing	*t*	*p*
Reference group (*n* = 45)	28.29 ± 0.64	18.69 ± 0.32	90.00	<0.001
Test group (*n* = 45)	28.31 ± 0.65	10.09 ± 1.14	93.14	<0.001
*t*	0.147	48.722		
*p*	0.883	<0.01		

**Table 7:** Average cost of PICC pipeline maintenance for one month of observation and nursing.

Group	PICC average cost of pipeline maintenance (yuan)
Reference group (*n* = 45)	216.78 ± 21.15
Test group (*n* = 45)	101.39 ± 10.37
*t* value	61.339
*p* value	<0.01

**Table 8:** To observe the incidence of PICC-related complications after one month of nursing.

Group	Phlebitis (example/%)	Percolation fluid at puncture point (example/%)	Catheter blockage (example/%)	Skin allergy (case/%)	Venous thrombosis (case/%)	Catheter prolapse (example/%)	PICC incidence of related complications (case/%)
Reference group (*n* = 45)	2/4.44	2/4.44	2/4.44	1/2.22	1/2.22	2/4.44	10/22.22
Test group (*n* = 45)	1/2.22	0/0.00	1/2.22	0/0.00	0/0.00	1/2.22	3/6.66
*χ* ^2^ value							4.405
*p* value							0.036

**Table 9:** The score of NSNS scale before nursing and 1 month after nursing.

NSNS scale score (points)	Before nursing	After one month of nursing	*t* value	*p* value
Reference group (*n* = 45)	78.19 ± 3.77	81.77 ± 4.21	4.249	≤0.001
Test group (*n* = 45)	78.21 ± 3.79	89.88 ± 5.01	12.461	≤0.001
*t* value	0.025	8.313		
*p* value	0.980	≤0.01		

## Data Availability

No data were used to support this study.
